# Comparison of Two Stump Closure Techniques in Laparoscopic Appendicectomy: A Single-Centre Prospective Cohort Study

This article has been retracted.

**DOI:** 10.7759/cureus.21796

**Published:** 2022-01-31

**Authors:** Ashwin Vinod, Binoj ST, Nivedita S Nanda, Greeshma C Ravindran

**Affiliations:** 1 General Surgery, Amrita Institute of Medical Sciences and Hospital, Kochi, IND; 2 Gastrointestinal Surgery, Amrita Institute of Medical Sciences and Hospital, Kochi, IND; 3 Biostatistics, Amrita Institute of Medical Sciences and Hospital, Kochi, IND

**Keywords:** cost analyses, hem-o-lok clip, endoloop, laparoscopic appendicectomy, uncomplicated appendicitis

## Abstract

Introduction

Acute appendicitis is a frequent illness that manifests as an emergency and most of the cases necessitate surgical intervention. One of the most critical processes in a laparoscopic appendicectomy is the closure of the appendicular stump. For the closure of the stump of the appendix, several approaches have been employed and explored, but the one with the best outcomes has yet to be proved. The purpose of this study was to evaluate the medical results and cost analyses of laparoscopic appendicectomy with two of the commonly used stump closure techniques - ENDOLOOP^®^ and Hem-o-lok^®^.

Materials and methods

A two-year prospective hospital-based cohort study was conducted from June 2019 to July 2021. All the patients in the study were randomly assigned to one of two experimental arms (ENDOLOOP^®^ and Hem-o-lok^®^). The clinical and follow-up data of these patients were collected and tabulated into a data sheet and analyzed.

Results

In total, 180 individuals were included in the research (90 in each arm). No statistically significant difference was found in comparing the age, gender or diameter of the appendix among the two groups. The time taken for surgery showed significant differences among the two study groups. The time taken for the procedure in the Hem-o-lok® group was significantly lower than the ENDOLOOP® group (40.3 ± 12.3 minutes vs 50.83 ± 10.5 minutes, p < 0.001). No intraoperative or immediate postoperative complications were noted in either of the groups. The average duration of hospital stay was 2.7 ± 0.9 days in the Hem-o-lok® group, while it was 3.1 ± 0.8 days in the ENDOLOOP® group (p = 0.986). The material cost for the stump ligation with Hem-o-lok® was Rs. 310 ± Rs. 76 while that using ENDOLOOP^®^ was Rs. 630 ± Rs. 118 (p < 0.001). In the Hem-o-lok^®^ subset of patients, the mean direct expenses of laparoscopic appendicectomy were considerably lower. During the 12-week follow-up period, none of the patients had any post-operative complications.

Conclusion

According to the results of this study, both the technical variations of appendix stump closure are equal in terms of postoperative complications. When compared to the ENDOLOOP^®^ group, the Hem-o-lok® group had a shorter duration of surgery and ended up spending less money. Hem-o-lok® clips have the potential to become the preferred way of anchoring the appendix base during laparoscopic appendicectomy.

## Introduction

Acute appendicitis is a frequent illness that manifests as an emergency and most of the cases necessitate surgical intervention. Laparoscopic appendicectomy is an effective surgical option for the treatment of these patients and helps in lowering hospital stay, post-surgical problems or discomfort as well as improving cosmesis and allowing for an early recovery [1,2]. One of the most critical processes in a laparoscopic appendicectomy is the closure of the appendicular stump, so as to minimise significant postoperative problems. Intracorporeal knotting needs strong surgical competence and the proper placement of a secure knot can be difficult at times, even in the hands of an experienced surgeon. Hence, the ligation of the appendix base can be quite challenging during laparoscopic appendicectomy. As a result of this problem, doctors are looking at several options for ligating the appendicular stump laparoscopically.

The best approach for sealing the stump during laparoscopy should be simple to use, safe, accessible, and dependable, with a shorter operating time and lower costs [2]. This is why many procedures for ligating the appendicular stump have been created, explored, and employed [3]. ENDOLOOP® metal endoclips, endo-stapler, harmonic or bipolar endocoagulation, Hem-o-lok® clips, and intracorporeal suture can all be used to ligate the appendicular stump during laparoscopic appendicectomy [2,4].

The cost of each medical or surgical operation is constantly evaluated in the present environment of ever-increasing healthcare expenditures. Methods to reduce costs and improve the quality of care provided to patients are continually being researched. One major strategy to raise the value of care is to find new ways to obtain identical results at a cheaper cost. The materials and instruments utilised are the most expensive aspects of any surgery. The choice of equipment and materials for every procedure in the field of minimal access surgery is determined by the operating surgeon's preference, expertise, and what instruments are available at that specific facility. Standardising instruments and improving the design of instruments for an easier learning curve have been sought to save expenses in laparoscopy.

Other alternatives include using less costly devices to achieve the same results as a more expensive surgical setup. Hem-o-lok® is a polymer clip that is used in a variety of laparoscopic operations, including cholecystectomy, nephrectomy, and other vascular procedures [2,5]. The purpose of this study was to compare the benefits and drawbacks of Hem-o-lok® against ENDOLOOP® for stump closure during laparoscopic appendicectomy, with respect to surgical cost, operating time, intraoperative complications, and postoperative problems.

## Materials and methods

A two-year prospective cohort study was conducted in the departments of General Surgery and Gastrointestinal Surgery at our tertiary care hospital in South India, from June 2019 to July 2021. The study was conducted following the ethical standards of the institutional research committee and with the 1964 Helsinki declaration and its later amendments. The data were collected after obtaining ethical clearance from the Institutional Research Board (ECASM-AIMS-2021-296). Informed consent had been obtained from all patients as a routine at admission for their enrolment into a study and for subsequent use of the data.

Inclusion criteria

Patients above the age of 18 years presenting to the departments of General and Gastrointestinal surgery with a clinical diagnosis of uncomplicated appendicitis, who are planned for elective laparoscopic appendicectomy.

Exclusion criteria

All patients with complicated appendicitis, as well as those not willing for laparoscopic appendicectomy or with a high risk of conversion to open appendicectomy.

Preoperative evaluation and management

Patients were started on empirical antibiotics and fluid maintenance prior to surgery. Abdominal ultrasonography was performed preoperatively (on an OPD basis or after admission) to confirm the diagnosis. Routine preoperative investigations were done, including routine blood tests, urine analysis, 12 lead ECG and a chest x-ray. After obtaining clearance from the anaesthesia team and any other concerned department in view of any underlying comorbidities, patients were planned for surgery on the following day.

Sample allocation

The patients were categorised into two groups, with sequential allocation used for sampling, with 90 patients in each research arm (Hem-o-lok® vs ENDOLOOP®)

Standard surgical technique followed using Hem-o-lok® clips

After receiving general anaesthesia, the patient was placed in a supine position and parts were painted and draped under stringent aseptic conditions. Transumbilical or infra umbilical incisions were used to introduce a 10-mm optical port. Following the principles of triangulation, a 5-mm trocar is placed at the LIF and another above the pubic region. The meso-appendicular window is generated once the appendix is recognised. The appendicular artery is cauterised, and the appendix is isolated at its base. Change the camera to a 5-mm scope and insert it into the LIF port. Using the Hem-o-lok® applicator and the 10 mm port, the base of the appendix is ligated with Hem-o- lok clips (Figure 1A). A second clip is inserted and put over the appendix's base (Figure 1A). Sometimes, an additional clip may be inserted at the appendix stump if the placement of the first clip is deemed to be defective or not secure (Figure 1B). The specimen is delivered through the 10 mm trocar after the appendicular base is transacted between the two clips. The sheath is closed using 1 - 0 polyglactin sutures, and the skin closure is done with 4 - 0 poliglecaprone subcuticular sutures.

**Figure 1:** Intraoperative image showing the application of Hem-o-lok clips during laparoscopic appendicectomy (A) Using the Hem-O-Lok® applicator, the base of the appendix is ligated with a Hem-o-lok clip and a second clip is inserted slightly away from the base. (B) An additional clip is placed at the base of the appendix, due to improper application of the first clip.

Standard surgical technique followed using ENDOLOOP®

After receiving general anaesthesia, the patient was placed in a supine posture and parts were painted and draped under stringent aseptic conditions. A 10 mm trocar for the scope is introduced via an umbilical port, and the appendix is identified. Following the principles of triangulation, a 5 mm trocar is placed at the LIF and above pubic regions, for creating the meso-appendicular window. The appendicular artery is cauterised and the appendicular base is ligated with an ENDOLOOP® (Figures 2A, 2B). A second ENDOLOOP® is put above the previous knot. The appendicular base is transacted between the two knots and delivered via the 10 mm trocar. The sheath is closed using 1 - 0 polyglactin sutures, and the skin closure is done with 4 - 0 poliglecaprone subcuticular sutures.

**Figure 2:** Intraoperative image showing the application of ENDOLOOP sutures during laparoscopic appendicectomy (A) Appendix passed through the ENDOLOOP suture. (B) ENDOLOOP suture tightened and secured at the base of the appendix.

Statistical analysis

The medical records of the patients included in the study were reviewed and the data so collected were tabulated into a data sheet. Statistical analysis was done using IBM SPSS version 20.0 (SPSS Inc, Chicago, IL, USA). For all the continuous variables, the results are given in Mean ± SD, and for categorical variables as a percentage. The mean difference in the numerical variables between groups was compared using the independent two-sample ‘t’-test for parametric data. To find out the association between two categorical variables, a chi-square test was applied.

## Results

In the period from June 2019 to July 2021, among the patients that presented to our hospital with appendicitis, laparoscopic appendicectomy was done for 373 patients. Among these patients, 180 patients that met our inclusion criteria were included in our study and allocated into the two study groups (90 in each study group). The various parameters compared in the two groups are shown in Table 1.

**Table 1:** Comparison of various parameters among the study groups

Variable	Hem-o-Lok Group	ENDOLOOP Group	P-value
Age (years)			
18-25	20 (22.2%)	21 (23.3%)	0.139
26-35	41 (45.5%)	38 (42.2%)	
36-45	16 (17.7%)	19 (21.11%)	
>45	13 (14.4%)	12 (13.33%)	
Mean Age (Years)	32.4 ± 5.7	34.9 ± 4.9	0.142
Gender			
Male	52 (57.7%)	53 (58.8%)	0.491
Female	38 (42.3%)	37 (41.2%)	
Duration of Surgery			
<45 mins	52 (57.7%)	10 (11.2%)	<0.001
45 mins-1 hour	32 (35.7%)	71 (78.8%)	
> 1 hour	6 (6.6%)	9 (10%)	
Mean Diameter of Appendix	9.73 mm ± 2.9 mm	9.93 mm ± 1.9 mm	0.337
Mean Duration of Surgery	40.3 ± 12.3 minutes	50.83 ± 10.5 minutes	<0.001
Mean Duration of Hospital Stay	2.7 ± 0.9 days	3.1 ± 0.8 days	0.986
Mean Material Cost	Rs. 310 ± Rs. 76	Rs. 630 ± Rs. 118	<0.001
Complications	Nil	Nil	

The mean age of the patients Hem-o-lok® group was 32.4 years ± 5.7 years while that in the ENDOLOOP® group was 34.9 years ± 4.9 years. Both groups showed a male preponderance (57.7% in Hem-o-lok® group and 58.8% in ENDOLOOP® group). There was no statistically significant difference in age or gender in comparing the two groups. Similarly, no statistically significant difference was found in the mean diameter of the appendix among the two groups (9.73 mm ± 2.9 mm vs 9.93 mm ± 1.9 mm).

The mean ± standard deviation of the duration of surgery in the Hem-o-lok® group was 40.3 ± 12.3 minutes, whereas that in the ENDOLOOP® group was 50.83 ± 10.5 minutes (p < 0.001). For further analyses, the patients were divided into 3 groups based on the duration of surgery ( <45 minutes, 45 minutes to 1 hour and >1 hour). On comparing the time taken for surgery, 57.7% patients in the Hem-o-lok® group were operated in less than 45 minutes, 35.7% took 45 minutes to an hour to complete, while 6.6% took more than an hour; and 78.8% patients in the ENDOLOOP® group were operated in the 45 minutes to 1-hour range, 10.3% were operated in less than 45 minutes, and 10% were operated in more than 1 hour. The difference in duration of surgery was statistically significant (p < 0.001).

The hospital material store was used to get the ENDOLOOP® and Hem-o-lok® clips. Patients were charged from the operation room based on the number of materials used. The material cost for the stump ligation with Hem-o-lok® was Rs. 310 ± Rs. 76 while that using ENDOLOOP® was Rs. 630 ± Rs. 118. The overall difference in the cost of materials and hence the cost of stump closure was found to be statistically significant (p < 0.001).

No intraoperative or immediate postoperative complications were noted in either of the groups. The average duration of hospital stay was 2.7 ± 0.9 days in the Hem-o-lok® group, while it was 3.1 ± 0.8 days in the ENDOLOOP® group (p = 0.986). During the 12-week follow-up period, none of the patients had any post-operative complications.

## Discussion

One of the most common general surgical diseases to be treated as an emergency is acute appendicitis [1,2]. Since the development of laparoscopic surgery, doctors have worked tirelessly to improve diagnostic procedures, develop multiple scoring systems, and discover new surgical techniques to minimise costs and shorten hospital stays for acute appendicitis treatment. To ligate the appendicular stump, many surgeons now utilise ENDOLOOP® or endostaplers [2].

ENDOLOOP® as well as endostaplers have a high safety quotient but the high cost of endostaplers and the high technical demand of ENDOLOOP® have forced the surgeons to look for even better alternatives. The use of Hem-o-lok® for stump closure is comparatively easier leading to a decreased surgical time and overall cost of the surgery. Different sizes of Hem-o-lok® clips are available (ranging from small to extra-large), of which the large clips (5-13 mm) were used in our study [2].

The patients in our study had similar age as well as similar gender distribution, comparable to various previous studies [2,6]. Our study showed an average diameter of 9.73 mm ± 2.9 mm in Hem-o-lok® group and 9.93 mm ± 1.9 mm in the ENDOLOOP® group. This was similar to a study conducted by Sik et al., which showed the mean diameter of the appendix in the Hem-o-lok® group to be 9.9 mm and 9.7 mm in the ENDOLOOP® group [2,7].

The time taken for surgery showed significant differences among the two study groups. Most of the patients operated on with Hem-o-lok® (57.7%) were operated on in less than 45 minutes while a majority of the patients operated on with ENDOLOOP® (88.8%) took more than 45 minutes. The average duration of surgery for the Hem-o-lok® group (40.3 ± 12.3 minutes) was significantly lower than the ENDOLOOP® group (50.83 ± 10.5 minutes). In a previous study conducted by Colak et al., the operating time in the Hem-o-lok® group was 64.7 minutes, while the operating time in the ENDOLOOP® group was 75.4 minutes, indicating that the Hem-o-lok® group had a shorter operating time. However, this difference was not statistically significant (p = 0.072) [8]. According to another study done by Delibegovic et al., the operational time in the Hem-o-lok® group was 47.1 minutes and in the ENDOLOOP® group was 38.7 minutes, indicating that the Hem-o-lok® group had a statistically significant shorter operating time (p < 0.001) [9].

According to the standard surgical technique used at our institution, only a single clip was applied at the base of the appendix and one clip with the specimen [2]. The overall ‘clips per patient’ ratio were 2.17 (owing to the small number of reapplication of clips). A study done by Partecke et al. advocated the use of a single clip at the base during laparoscopic appendicectomy [10]. The results were similar to the previous studies, thus adding strength to the existing literature [10].

The cost of surgery showed a considerable decrease in the Hem-o-lok® group as compared to the ENDOLOOP® group (Rs. 310 ± Rs. 76 vs Rs. 630 ± Rs. 118). This was similar to the observations in the study conducted by Colak et al. ($30 in Hem-o-lok® group vs $120 in ENDOLOOP® group) [8].

There were no postoperative complications in our study, such as appendicular abscess, cutting through the appendicular base, leak, fistula formation or post-operative discomfort. In a study conducted by Soll et al., it was found that using non-absorbable Hem-o-lok® clips to ligate the appendicular stump resulted in a lower incidence of intra-abdominal surgical abscesses than with ENDOLOOP® [11]. Samir Delibegovic et al. published two trials in 2009 and 2012 that found no intraoperative or postoperative problems, comparable to ours [9,12].

Multiple studies looked at the safety of using Hem-o-lok® and ENDOLOOP® to ligate the appendicular base during laparoscopic appendicectomy [13,14]. ‘Hem-o-lok® may be utilised safely in various laparoscopic surgeries provided the right technique is mastered’, Aminian et al. concluded [15]. In our study, none of the patients who had laparoscopic appendicectomy experienced any intraoperative or postoperative problems, demonstrating that Hem-o-lok® clips are as safe as ENDOLOOP® for ligating the appendicular stump, with a lower material cost.

Limitations

Patients in the paediatric age group and those with complicated appendicitis were not included in the study. Also, the comorbidities of the patients in the study were not taken into account.

## Conclusions

Advanced laparoscopic training is difficult to come by in a developing nation like India. As a result, approaches with a low learning curve should be used in a variety of advanced laparoscopic operations. We believe that Hem-o-lok® will be a simpler procedure for novices to master, saving operating time. Hem-o-lok® is statistically cheaper than ENDOLOOP®, according to a cost comparison assessment and Hem-o-lok® surgery took less time on average. There were no intra-operative or post-operative problems in the Hem-o-lok® group. Hence, we advocate the use of Hem-o-lok® as a safe, simpler and cost-effective way to ligate an appendicular stump in uncomplicated laparoscopic appendicectomy.
